The article "High Prevalence of Drug Resistance in Animal Trypanosomes without a History of Drug Exposure" was published in 2011. Journal: PLoS Negl Trop Dis.

# High Prevalence of Drug Resistance in Animal Trypanosomes without a History of Drug Exposure

**DOI:** 10.1371/journal.pntd.0001454

**Published:** 2011-12-20

**Authors:** Simbarashe Chitanga, Tanguy Marcotty, Boniface Namangala, Peter Van den Bossche, Jan Van Den Abbeele, Vincent Delespaux

**Affiliations:** 1 Institute of Tropical Medicine Antwerp, Antwerp, Belgium; 2 Department of Paraclinical Studies, School of Veterinary Medicine, University of Zambia, Lusaka, Zambia; 3 Department of Veterinary Tropical Diseases, University of Pretoria, Onderstepoort, South Africa; Swiss Tropical and Public Health Institute, Switzerland

## Abstract

**Background:**

Trypanosomosis caused by *Trypanosoma congolense* is a major constraint to animal health in sub-Saharan Africa. Unfortunately, the treatment of the disease is impaired by the spread of drug resistance. Resistance to diminazene aceturate (DA) in *T. congolense* is linked to a mutation modifying the functioning of a P2-type purine-transporter responsible for the uptake of the drug. Our objective was to verify if the mutation was linked or not to drug pressure.

**Methodology/Principal Findings:**

Thirty-four *T. congolense* isolates sampled from tsetse or wildlife were screened for the DA-resistance linked mutation using *Dpn*II-PCR-RFLP. The results showed 1 sensitive, 12 resistant and 21 mixed *Dpn*II-PCR-RFLP profiles. This suggests that the mutation is present on at least one allele of each of the 33 isolates. For twelve of the isolates, a standard screening method in mice was used by (i) microscopic examination, (ii) trypanosome-specific 18S-PCR after 2 months of observation and (iii) weekly trypanosome-specific 18S-PCR for 8 weeks. The results showed that all mice remained microscopically trypanosome-positive after treatment with 5 mg/kg DA. With 10 and 20 mg/kg, 8.3% (n = 72) and 0% (n = 72) of the mice became parasitologically positive after treatment. However, in these latter groups the trypanosome-specific 18S-PCR indicated a higher degree of trypanosome-positivity, i.e., with a unique test, 51.4% (n = 72) and 38.9% (n = 72) and with the weekly tests 79.2% (n = 24) and 66.7% (n = 24) for 10 and 20 mg/kg respectively.

**Conclusion/Significance:**

The widespread presence of the DA-resistance linked mutation in *T. congolense* isolated from wildlife suggests that this mutation is favourable to parasite survival and/or its dissemination in the host population independent from the presence of drug. After treatment with DA, those *T. congolense* isolates cause persisting low parasitaemias even after complete elimination of the drug and with little impact on the host's health.

## Author Summary

Trypanosomosis is responsible for the death of 3 million heads of cattle yearly, with 50 million animals at risk in sub-Saharan Africa. DA, a commonly used drug against the disease, was marketed decades ago. Drug resistance is reported in 21 African countries. A common argument about the origin of drug resistance is the selection by the drug of rare individuals that are naturally resistant and the propagation of those individuals in the population because of the competitive advantage they have when exposed to drug. When the drug pressure decreases, the wild-type individuals regain their supremacy. The principal objective of this study was thus to estimate the prevalence of trypanosomes resistant to DA in a population that was never exposed to the drug. Our results showing a high prevalence of drug resistance in environments free of any drug pressure is thought provoking and suggests that ceasing the use of DA will not allow for a return to a DA-sensitive population of trypanosomes. Drug resistance in animal trypanosomes thus present a pattern different from what is observed with *Plasmodium sp.* (causative agent of malaria) where a complete stoppage in the use of the chloroquine allows for a return to drug sensitivity.

## Introduction

Animal trypanosomosis is one of the major constraints to animal health and production in sub-Saharan Africa and has a major impact on people's livelihoods. The annual estimated direct and indirect losses due to the disease run into billions of dollars [1]. The fight against the disease is either managed by the control of the vector or of the parasite or a combination of both. However, in poor rural communities, which are mostly affected by the disease, control is mainly relying on the use of trypanocidal drugs [2]. The main drugs used by livestock keepers are isometamidium chloride (ISM) which has both curative and prophylactic effects and DA which has only curative properties. These drugs have been in use for more than half a century now. Geerts & Holmes [3] estimated that ∼35 million doses of trypanocides are administered every year in sub-Saharan Africa, with ISM, ethidium bromide and DA representing 40%, 26% and 33% respectively. Despite the high usage of these veterinary trypanocides, the interest of pharmaceutical industries to invest in research for developing new products remains low, leaving farmers to rely on the existing drugs. Due to the privatization of veterinary services in most parts of Africa, farmers have easy access to these trypanocides and this has resulted in rampant misuse and under-dosage of the medications, actions which have been blamed for the emergence of trypanocidal drug resistance [4], [5]. To date, there are 18 countries in which trypanocidal drug resistance has been reported [2] and more recently in Benin, Ghana and Togo (Réseau d'épidémiosurveillance de la résistance aux trypanocides et aux acaricides en Afrique de l'Ouest – RESCAO, unpublished data). However, most of these reports seem to be confined to areas where the disease is endemic [6]. Whilst reports of the occurrence of trypanocidal drug resistance are increasing, it is not really clear whether this is due to a real increase of the trypanocide resistance problem or just an increased interest by scientists [2]. However, a report by Delespaux *et al.* [7] of a five-fold increase in the prevalence of DA resistance over a seven year period in the Eastern Province of Zambia, suggests that there is indeed an aggravation of the phenomenon. Even more worrying are the recent reports of multiple drug resistance (to ISM and DA) [8] because this is threatening the last stand to overcome drug resistance through the use of the sanative pair. Here, the concept of the sanative pair recommends the use of two trypanocides (e.g. DA and ISM) unlikely to induce cross-resistance. The first drug is used until resistant strains of trypanosomes appear and then, the second is substituted and used until the resistant strains have disappeared from cattle and tsetse [9]. DA uptake is predominantly driven by a P2-type purine transporter (TbAT1) in *T. brucei* and a set of six point mutations in this gene has been shown to be linked with resistance to the veterinary drug DA [10]. However, Delespaux *et al.* [11] found that in *T. congolense* a single point mutation in an orthologous gene of the *T. brucei* P2-type purine transporter (TcoAT1) was correlated to resistance to DA in that species. Such genetic mutations conferring drug resistance in parasites are thought to arise randomly and to spread out when the parasite population is exposed to the drug because the mutation(s) is/are conferring a selective advantage compared to the wild type population [12]. Hastings [13] identified the following as some of the important factors determining the rate of evolution of the drug resistance in a parasite population: (i) the mutation rate from wild type to resistant genotype, (ii) the level and pattern of drug use and (iii) the parasitaemia within the host i.e. the number of parasites exposed to the drug after the treatment of the host. Genetic mutations can impair the fitness of parasites allowing a higher survival in presence of drugs but a progressive elimination in absence of drug pressure [14]. However, these mutations will still persist in a parasite population at low frequencies governed by the mutation-selection balance [15] with their proportion determined by the relative fitness of the mutant versus the wild type parasites [16]. Innate phenotypes resistant to DA and to homidium were already reported in *T. vivax* and *T. congolense* respectively [17], [18]. The objective of this study was thus to examine the prevalence of the mutation linked to DA resistance in natural *T. congolense* populations that never were exposed to the pressure of the drug, this prevalence being the result of the balance between the mutation rate and the ecological fitness of the mutated trypanosome.

## Materials and Methods

### Ethics statement

This is to certify that the experiments carried out at the Institute of Tropical Medicine in the framework of this study were approved by the Ethics Committee of the Institute of Tropical Medicine and that the study was conducted adhering to the institutional guidelines for animal husbandry. In Belgium, protection of experimental animals is regulated by the Royal Decision of 14 NOV 1993.

### Study areas and isolation of trypanosomes

All the trypanosomes used in this study were isolated in protected areas where game animals served as exclusive hosts for the trypanosomes. The study areas were the South Luangwa National Park in Zambia, Mana Pools National Park in Zimbabwe and the Hluhluwe-Umfolozi Game Reserve in the South African KwaZulu-Natal. In the South Luangwa National Park, tsetse flies (*Glossina morsitans morsitans* and *G. pallidipes*) were trapped using epsilon traps [19] and flies were dissected to determine their infection status. The mouthparts of tsetse flies, infected with trypanosomes in both the midgut and mouthparts, were injected intraperitoneally (I.P.) in an immunosuppressed mouse (300 mg/kg Cyclophosphamide, Endoxan®, Baxter S.A.). The inoculated mice were then monitored for the development of a trypanosome infection, with the parasitaemic blood collected from each positive mouse considered as an isolate. In the Hluhluwe-Umfolozi Game Reserve, isolation of the trypanosomes was completed from buffaloes belonging to herds that were selected randomly for tuberculosis testing. From each of the 132 buffaloes sampled, a volume of 0.3 ml of jugular blood was injected IP in two mice. The injected mice were then monitored for development of a trypanosome infection, with the parasitaemic blood collected from each positive mouse considered as an isolate. In the Mana Pools National Park, tsetse flies (*Glossina morsitans morsitans* and *G. pallidipes*) were trapped using epsilon traps [19] and flies were dissected to determine their infection status [20]. The mouthparts of those flies infected in both the midgut and mouthparts, were collected and preserved in a buffer of 0.5 M guanidine chloride, pH 8.

All 34 isolates that were collected belonged to the *T. congolense* Savannah sub-group as determined by the trypanosome specific 18S-PCR-RFLP [21]. The median survival times of mice inoculated with the isolates from Hluhluwe-Umfolozi Game Reserve and from the South Luangwa National Park, without treatment, are described by Van den Bossche et al [22].

### DA resistance genetic profiling by *Dpn*II-PCR-RFLP

DNA extraction was conducted for all the 34 strains collected. For the isolates that were successfully grown in mice, blood from one parasitaemic mouse was collected and trypanosome DNA extracted using the Gentra® extraction kit as according to manufacturer's recommendations. For those strains which were preserved in guanidine storage buffer, the trypanosome DNA was also extracted. Briefly, the mouthparts were removed from the buffer into 100 µl of grinding buffer (80 mM NaCl, 160 mM sucrose, 100 mM Tris-HCl pH 8.6, 60 mM EDTA and 0.5% SDS) and incubated at 65°C for one hour, with shaking. The dried pellet was then suspended in 40 µl of TE buffer and this was used for DNA analysis.

The *Dpn*II-PCR-RFLP was performed on the 34 isolates to check for the presence of the mutation in the P2-type purine transporter gene that is associated with resistance to DA [11]. The PCR and analysis of the amplicon was done using the method described by Vitouley et al [23] but without the whole genome amplification step. In brief, a standard PCR was conducted on DNA samples using the following primers (Ade2F ATAATCAAAGCTGCCATGGATGAAG and Ade2R GATGACTAACAATATGCGGGCAAAG) and a Sigma thermocycler®.

### *In vivo* drug sensitivity testing (multi doses test in mice)

The method described by Eisler *et al.* [24] was used for evaluating the sensitivity of the isolates to DA. The method was slightly modified as follows: the 12 field isolates were tested at doses of 20 and 10 mg/kg DA administered intraperitoneally. Inoculation of the trypanosomes, monitoring of the infected mice and interpretation of the results was done as described by Eisler *et al.* [24]. Briefly, 10^5^ trypanosomes were inoculated in each mouse and treatment was administered 24 hours after inoculation. For each of the 12 isolates, two groups of six mice were used for each drug dosage and its control. An isolate was considered resistant to a particular dose if at least two of the six mice in that treatment group relapsed (assessed by microscopical examination). At the end of the 60 days experimental period, tail blood from all mice was spotted onto a Whatman® Nr 4 filter paper and examined using the trypanosome specific 18S-PCR [21] to detect presence of trypanosomes that could not be detected by the microscopical examination. Mice were euthanized at the end of the examination period. A reference strain sensitive to DA (TRT8) was added as quality control for the trypanocide used. This isolate originates from cattle in the Eastern Province of Zambia and was then cloned visually from a single trypanosome. It shows a *T. congolense* savannah type profile with the trypanosome specific 18S-PCR-RFLP and a DA-sensitive profile with *Dpn*II-PCR-RFLP.

### Monitoring trypanosome presence by PCR

To determine the presence of trypanosomes in mice treated with DA at a dose of 10 or 20 mg/kg, blood samples of the mice infected with the 4 different isolates (MF2, MF3, MF4, MF5 and TRT8 as the sensitive control) were weekly spotted on a Whatman® Nr 4 filter paper for 8 weeks and examined by the trypanosome specific 18S-PCR to detect the presence of trypanosomes. Proportions of relapses were calculated on the basis of 24 mice leaving the sensitive control (TRT8) out.

### Degradation of trypanosomal DNA in vivo

Blood (1.4 ml) was collected from a highly parasitaemic mouse (10^8^ trypanosomes/ml blood) and DNA extraction was done using a Gentra® extraction kit for a final volume of 200 µl of DNA solution. 100 µl of this solution was intravenously injected into each of two mice. Tail blood was then collected on filter paper 30 min. and 1, 3, 6, 7, 13, 15, 16, 21 & 28 days after the injection and examined by the trypanosome specific 18S-PCR to detect the presence of trypanosome DNA.

## Results

Six isolates were collected in the South Luangwa National Park, 6 in the Hluhluwe-Umfolozi Game Reserve and 22 from Mana Pools National Park. One strain showed a sensitive *Dpn*II-PCR-RFLP profile, 12 showed a resistant profile whilst the remaining 21 showed a mixed profile. When a mixed profile is observed, a heterozygous trypanosome population cannot be differentiated from a mixture of homozygous sensitive and resistant trypanosomes as the experimental material are isolates and not cloned trypanosomes.

The results of the drug sensitivity tests in mice are summarized in table 1. This was done only for the 12 isolates isolated from South Luangwa National Park and Hluhluwe-imfolozi game reserve since only those had been successfully grown in mice. Using the methodology and criteria described by Eisler et al. (2001) only one resistant isolate was identified in the group treated with 10 mg/kg and none in the group treated with 20 mg/kg. However, using the more sensitive trypanosome-specific 18S-PCR once at the end of the observation period, more trypanosome-positive mice were observed in these groups, with 51.4% (n = 72) and 38.9% (n = 72) positive PCR results respectively. At a dose of 5 mg/kg, all mice relapsed based upon microscopic examination as well as PCR.

**Table 1:** *Dpn*II-PCR-RFLP-profiles of the different wild *T. congolense* strains and their drug sensitivity status in infected mice treated with 20 and 10 mg/kg diminazene (DA).

		10 mg/kg DA		20 mg/kg DA	
Strain	Profile	Mic. +	PCR +	Mic. +	PCR +
MF 1	R	0/6*	5/6	0/6	1/6
MF 2	R	0/6	1/6	0/6	3/6
MF 3	R	5/6	6/6	0/6	1/6
MF 4	M	1/6	5/6	0/6	5/6
MF 5	R	0/6	1/6	0/6	2/6
MF 6	R	0/6	2/6	0/6	2/6
BT0106	M	0/6	4/6	0/6	5/6
BT0206	M	0/6	3/6	0/6	5/6
BT0306	M	0/6	3/6	0/6	3/6
BT0306 ISM	R	0/6	4/6	0/6	3/6
BT0406	M	0/6	3/6	0/6	1/6
BT0506	R	0/6	0/6	0/6	1/6
*TRT8 sensitive control*	*S*	*0/6*	*0/6*	*0/6*	*0/6*
**CRS**		**8.33%**	**51.38%**	**0%**	**38.88%**

This drug sensitivity status was scored for each individual mouse by microscopy and trypanosome specific 18S-PCR analysis, 60 days after the initial treatment. With R for resistant, M for mixed, S for sensitive, CRS for cumulative relapsing rate and *for number of mice positive by the trypanosome specific 18S-PCR.

When considering the weekly follow up, the parasitaemias of the groups inoculated with the 4 isolates (MF2, MF3, MF4 & MF5) were intermittent throughout the period of observation and the cumulative amount of relapses was impressive with 79.2% (n = 24) and 66.7% (n = 24) in the groups treated with 10 and 20 mg/kg respectively. As an example, the results for the weekly evolution of parasitaemia as determined by trypanosome specific 18S-PCR post-treatment with 20 mg/kg DA are shown in table 2.

**Table 2:** Weekly evolution of the parasitaemia as determined by the trypanosome specific 18S-PCR post-treatment with 20 mg/kg.

Strain	W1	W2	W3	W4	W5	W6	W7	W8	CR
MF 2	2/6*	3/6	2/6	2/6	2/6	0/6	2/6	2/6	5/6
	(1,5)**	(1,5,6)	(3,5)	(1,6)	(1,2)	(-)	(2,6)	(2,5)	
MF 3	0/6	1/6	1/6	0/6	1/6	1/6	1/6	2/6	2/6
	(-)	(1)	(1)	(-)	(3)	(1)	(1)	(1,3)	
MF 4	0/6	2/6	2/6	0/6	1/6	1/6	0/6	1/6	3/6
	(-)	(1,3)	(2,3)	(-)	(3)	(1)	(-)	(2)	
MF5	0/6	3/6	5/6	0/6	3/6	2/6	3/6	5/6	6/6
	(-)	(1,5,6)	(1,2,3,5,6)	(-)	(2,5,6)	(2,4)	(2,4,5)	(1,3,4,5,6)	
*TRT8 SC*	*0/6*	*0/6*	*0/6*	*0/6*	*0/6*	*0/6*	*0/6*	*0/6*	*0/6*
	*(-)*	*(-)*	*(-)*	*(-)*	*(-)*	*(-)*	*(-)*	*(-)*	
**Total CR**									**66.66%**

With TRT8 SC as sensitive control, Wx for week number; CR for cumulative relapses, *for number of mice positive using the trypanosome specific 18S-PCR and **for ID number of the 18S-PCR positive mice.

Finally, the DNA of trypanosomes, when injected intravenously into mice, persisted in the blood for 14 days beyond which it was no longer detectable by the trypanosome specific 18S-PCR.

## Discussion

The high prevalence of the mutation in the genes coding for P2-type purine transporters in *T. congolense* populations that were never exposed to any drug pressure is thought provoking. The correlation of this mutation with phenotypic resistance to DA is largely demonstrated by the multi-dose sensitivity testing in mice [25]. This high prevalence of the mutation conferring resistance to DA was not expected in regions where the circulating trypanosome populations were never exposed to any trypanocidal drug pressure. Indeed, mutations conferring drug resistance are often related to a fitness cost for the parasite and are supposed to be selected out in the absence of drug as it is described, for example, in malaria parasites [14], [15]. On the contrary, a complete stoppage of the use of DA would not allow for a return to a DA-sensitive population of trypanosomes.

The observed high prevalence of the DA-resistance linked mutation (97.1%) in the wild *T. congolense* populations suggests that it confers a selective advantage over the non-mutated strains and that it is part of the normal genotypic diversity of a wild trypanosome population. However, the observation of 97.1% of mutated strains is in contrast with previous studies in Eastern Province of Zambia reporting 38.5% of mutated strains in 1996. Interestingly, without any change in the drug use this proportion already raised to 89.5% seven years later, in 2004. This situation and trend to an increasing percentage of the mutated strains might be the result of the massive, systematic and widespread ISM block treatments that were organized in the eighties by the Zambian government in an attempt to eradicating trypanosomes from tsetse flies [26]. This massive treatment campaign presumably resulted in a severe genetic bottleneck in the existing *T. congolense* population constituting mainly of non-mutated strains (for DA). This scenario could have simply occurred by a random effect on the selection. At the end of the massive drug pressure, we can reasonably assume that the trypanosome population multiplied again and that the percentage of mutated strains increased gradually due to a fitness advantage of the mutated strains.

Albeit the microscopical examination failed to detect nearly all relapses except after treatment at 5 mg/kg DA, the results of the trypanosome specific 18S-PCR confirms unequivocally the numerous relapses after treatment at 10 and 20 mg/kg. This PCR-positivity is not due to persistent circulating trypanosomal DNA as we demonstrated that injected DNA of trypanosomes is no longer PCR-detectable in the mouse blood circulation 14 days after the initial injection. This strongly suggests that the positive PCR results observed in the microscopically negative mice indicates the presence of living trypanosomes circulating at low abundance. With a single examination at the end of the observation period, more than one half and one third of the isolates relapsed at 10 and 20 mg/kg respectively. Furthermore, the weekly follow up of the parasitaemias shows clearly that the increased frequency of observation after treatment (8 rather than 1 at the end of the observation period) raises the observed relapses rate to 79.2% and 66.7% for 10 and 20 mg/kg respectively. Remarkably, the positive outcome of the trypanosome specific 18S-PCR tests done two months after treatment compared to the negative microscopical examinations suggests that the relapsed trypanosome populations remain at very low densities. This is surprising since it can be assumed that no active DA is circulating in the blood two months after the treatment. Indeed, the recommended withdrawal time prior slaughtering for livestock is 21–35 days and the elimination rate of DA is not expected to be longer in rodents as it is a smaller species with a higher metabolism [27], [28]. This observation seems to suggest that the DA treatment has reduced the impact of the relapsed trypanosome infection on its host. This becomes evident when observing the median survival time of the mice that are infected with the same isolates before DA treatment [22]. Without treatment, 50% and 67% of the mice die within 10 and 20 days respectively. The predicted median survival time for the two less virulent isolates is 24 and 51 days. None of the mice is expected to survive for 60 days as they manage in good shape in our drug resistance test. The development of such cryptic infections could be due to the effect of the drug reducing the parasitaemia to a level low enough for host immunity to maintain the parasites at a very low density. If this observation can be confirmed in livestock, it would drastically change the rationale of treatment guidelines in case of DA resistance.

Those very low parasitaemias with very limited impact on the host induced by the DA treatment are interesting. Similar results were obtained in cattle when experimentally infected with ISM resistant strains and treated with ISM at the first peak of parasitaemia. The impact of the infection on the PCV was not very pronounced (average PCV reduction 8 to 14 weeks after treatment: 5.9%; 95% CI: 4.5–7.3) [29].

Our findings have important repercussions for the understanding of the epidemiology of trypanocidal drug resistance in livestock trypanosomosis and its control: (i) considering the high prevalence of the resistant genotype in the natural *T.congolense* isolates from Zambia and South Africa, development of resistance to DA once these strains are circulating in livestock seems to be unavoidable and quick, (ii) regular under-dosing will support the spread of the resistant wild genotypes in the livestock population [4], [26] and finally (iii) if our results are further confirmed in livestock, the advice could be to continue treating cattle even in the presence of drug resistance as the treatment would allow the host to control the parasite and the corresponding disease at an acceptable level.
